# Deep Learning-Based Methods for Sentiment Analysis on Nepali COVID-19-Related Tweets

**DOI:** 10.1155/2021/2158184

**Published:** 2021-11-01

**Authors:** C. Sitaula, A. Basnet, A. Mainali, T. B. Shahi

**Affiliations:** ^1^Department of Electrical and Computer Systems Engineering, Monash University, VIC, Clayton, 3800, Australia; ^2^Central Department of Computer Science and Information Technology, Tribhuvan University, Kathmandu 44600, Nepal; ^3^Kist College, Kathmandu, Nepal; ^4^Aryan School of Engineering, Kathmandu, Nepal; ^5^School of Engineering and Technology, Central Queensland University, Rockhampton, QLD 4701, Australia

## Abstract

COVID-19 has claimed several human lives to this date. People are dying not only because of physical infection of the virus but also because of mental illness, which is linked to people's sentiments and psychologies. People's written texts/posts scattered on the web could help understand their psychology and the state they are in during this pandemic. In this paper, we analyze people's sentiment based on the classification of tweets collected from the social media platform, Twitter, in Nepal. For this, we, first, propose to use three different feature extraction methods—fastText-based (ft), domain-specific (ds), and domain-agnostic (da)—for the representation of tweets. Among these three methods, two methods (“ds” and “da”) are the novel methods used in this study. Second, we propose three different convolution neural networks (CNNs) to implement the proposed features. Last, we ensemble such three CNNs models using ensemble CNN, which works in an end-to-end manner, to achieve the end results. For the evaluation of the proposed feature extraction methods and CNN models, we prepare a Nepali Twitter sentiment dataset, called NepCOV19Tweets, with 3 classes (positive, neutral, and negative). The experimental results on such dataset show that our proposed feature extraction methods possess the discriminating characteristics for the sentiment classification. Moreover, the proposed CNN models impart robust and stable performance on the proposed features. Also, our dataset can be used as a benchmark to study the COVID-19-related sentiment analysis in the Nepali language.

## 1. Introduction

Sentiment analysis is the process of identifying the polarity of documents into different classes, such as positive, negative, and neutral. It has a wider range of application areas such as opinion mining, recommendation systems, and health informatics. Based on the opinion of people, businesses make strategic plans to improve their services, thereby increasing profits. Similarly, based on the analysis of tweets, people can assess human psychology and their behaviors, which are linked to their health status. For the sentiment analysis, researchers have been using different kinds of textual documents such as Facebook posts and tweets. In this study, we study recent COVID-19 tweets related to sentiment classification works around the world. However, there are no such existing works in Nepali language to this date.

Existing works [2–14] related to COVID-19 tweets' analysis in other languages apart from the Nepali language not only underscore the efficacy of sentiment analysis but also support the role of traditional machine learning and deep learning algorithms on sentiment analysis tasks. In most of these works, they prefer using deep learning-based methods for sentiment analysis. Similarly, regarding the analysis of such tweets, researchers are also focusing on different aspects such as topic modeling and sentiment classification. Here, they prefer using the syntactic-based feature representation methods such as Term-Frequency and Inverse Document-Frequency (TF-IDF) method mostly.

There are three main limitations in the aforementioned works. First, most of the existing works [2, 4, 5, 12] on COVID-19-related tweets are performed in high-resource languages such as English and Arabic. The approach used by high-resource language might be inapplicable to low-resource languages such as Nepali, which is based on Devanagari script and has 36 consonants (33 are distinct consonants and 3 are combined consonants), 13 vowels, and 10 numerals (Figure 1) [1, 15, 16]. Second, their investigation mainly targets either clustering the tweets into various themes/topics or classifying their polarity into three classes (negative, positive, or neutral) using the well-established feature extraction methods such as BERT, Word2Vec, and Glove. However, these feature extraction methods might be insufficient to capture the semantic information of textual documents or tweets written in the Nepali language. Third, existing methods [17, 18] capture the unimodal information only (e.g., bag-of-words using TF-IDF approach), which is insufficient to discriminate the complex tweets requiring the complementary semantic information (e.g., contextual) during classification. Also, their methods might not be appropriate to tweet dataset having a fewer number of tokens.

Given the limitations of existing works, we propose to use three kinds of feature extraction methods (fastText-based method, domain-specific method, and domain-agnostic method) for Nepali tweets' representation. First, with the help of the pretrained fastText-based method [19], we capture the semantic information. Here, it imparts a 300-D sized embedding vector for each word. Second, the domain-specific method helps to preserve the focused semantic information of the particular domain. For example, semantic features based on the COVID-19-related tweets could learn more informative features. For this, we employ the probabilistic feature extraction approach as suggested by Sitaula et al. [1] recently, which calculates the probability of each input word across all categories and finally and attains the feature vector depending on the number of categories present in the dataset. Last, with the help of the domain-agnostic method, we capture the semantic information using the cross-domain approach, which means that we transfer the knowledge to current COVID-19 domain from another domain such as news categories. For this, we follow a similar probabilistic approach as in the domain-specific method to extract this kind of feature. Furthermore, given the prominent classification abilities of deep learning methods in natural language processing, we propose four different CNN models to carry out the sentiment analysis of COVID-19 tweets written in the Nepali language. The first CNN model is used to train the contextual information achieved from the pretrained fastText [19] model. The second CNN model is used to train the domain-specific feature vectors. The third CNN model is used to train the domain-agnostic feature vectors. Since three different CNN models yield three different decision scores based on the corresponding information for each tweet, we, finally, aggregate them to include all three information using the ensemble CNN model.

In summary, our paper has the following contributions:

- We prepare a public Nepali COVID-19 tweets' dataset, called NepCOV19Tweets, for COVID-19-related sentiment analysis in the Nepali language. This dataset can be used as a benchmark in Nepali COVID-19 tweets related to sentiment analysis research.
- To the best of our knowledge, this is the first work of sentiment analysis on Nepali COVID-19 tweets with three classes.
- We propose to use three different feature extraction methods—fastText-based feature extraction (ft), domain-specific probability-based (ds), and domain-agnostic probability-based (da) feature extraction—for the representation of tweets written in the Nepali language. Among these three methods, two methods (“ds” and “da”) are novel feature extraction methods used in this study.
- We propose three different CNN models for the sentiment classification of tweets using three different feature extraction methods based on fs, ds, and da, respectively. In addition, for the end results, we design an ensemble CNN model that captures the three different information on the fly.
- We validate our proposed methods against traditional machine learning methods and state-of-the-art methods on Nepali COVID-19 tweets' dataset (NepCOV19Tweets). The experimental results on such dataset show that our method produces a stable and promising classification performance.

The rest of this paper is organized as follows.  Section 2 studies the related works of COVID-19-related tweets' classification. Similarly, Section 3 explains the materials, proposed methods, and implementation. Furthermore, Section 4 discusses the results and compares them with the existing state-of-the-art methods, and Section 5 concludes the paper with limitations and future works.

## 2. Related Works

Under the COVID-19 tweets' analysis, several works have been carried out around the world [2–14] in a short span of time. Most of the research works are based on high-resource languages such as English.

Boon et al. [2] proposed a sentiment analysis and topic modeling study on COVID-19 tweets to increase the understanding of its trend and concern. They analyzed COVID-19-related 107,990 tweets extracted from 13 December to 9 March 2020. Their results indicate that the people have a negative outlook towards COVID-19 and express them into three different themes such as COVID-pandemic, Control, and Reports. Another work related to the classification of tweets into either positive or negative was carried out by Nemes et al. [3] using the recurrent neural network (RNN). They established their tweets' dataset based on COVID-19 with four fine-grained classes: weak positive, strong positive, weak negative, and strong negative. Their method outperforms TextBlob [22]. Furthermore, Manguri et al. [4] collected a seven-day tweets related to COVID-19 and performed sentiment analysis using TextBlob [22]. Their results show that 60% of tweets are about “smooth and relaxed,” whereas 13% of tweets are related to “feeling hopeful. ” On the other hand, only 7% are related to “relieved mood. ” Similarly, Naseem et al. [5] compared the traditional machine learning methods such as support vector machine (SVM), Naive Bayes (NB), decision tree (DT), random forest (RF), and deep learning methods such as convolution neural network (CNN), and bidirectional long short-term memory (BiLSTM), in combination with various embedding vectors such as fastText [19], Glove [23], and Word2Vec [24] on their COVID-19 tweets' datasets into three classes (negative, positive, and neutral). Their results depict that the deep learning (DL)-based methods outperform the traditional ML methods. They also conducted the fine tuning of the transformer-based learning methods, such as BERT [25], DistilBERT [26], XLNET [27], and ALBERT [28], where the highest accuracy of 92.90% was achieved by ALBERT.

Furthermore, Rustam et al. [7] compared the performance of five machine learning algorithms: random forest, extra tree classifier, XGBoost classifier, decision tree, and long short-term memory (LSTM) for COVID-19 tweet sentiment classification into three classes: positive, negative, and neutral. For this, they utilized two widely used feature extraction methods: Bag-of-Words (BOW) and Term-Frequency and Inverse Document Frequency (TF-IDF). Their results show that the extra tree classifier with an accuracy of 93.00% outperforms all remaining classifiers. In the meantime, Basiri et al. [8] proposed the ensemble deep learning method to classify tweets sentiment using five base learners: Naive Bayes support vector machine (NBSVM), CNN, BiGRU, FastText-based model, and DistilBERT-based model. Their results show that the stacked ensemble method outperforms all other methods with an accuracy of 85.8%. Similarly, Kaur et al. [9] created a dataset of COVID-19 tweets using five different hashtags such as “#COVID-19”, “#coronavirus,” “#deaths,” “#new case,” and “#recovered. ” They compared the performance of a hybrid heterogeneous support vector machine (SVM) with the recurrent neural network (RNN) for tweets' sentiment classification into three classes (positive, negative, and neutral). Their results show that SVM classifies more tweets into neutral class, whereas RNN categorizes more tweets into positive class. A long short-term memory (LSTM) model was employed by Imran et al. [11] to access the sentiment polarity of people from different cultures to the coronavirus using COVID-19-related tweets dataset, called Sentiment140. Their results show a higher correlation between the USA and Canada (0.96 for positive and 0.97 for negative sentiments) and between India and Pakistan (0.81 for positive and 0.86 for negative sentiments). However, a low correlation between Norway and Sweden (0.50 for negative and 0.40 for positive sentiments) exists. Furthermore, sentiment analysis on 13.9 million COVID-19-related tweets was conducted by Chandrasekaran et al. [12], which identified the trends and variations of COVID-19-related tweets, key topics, and associated sentiments before and after the pandemic. They inferred 26 topics on COVID-19-related tweets using latent Dirichlet analysis (LDA) and grouped them into 10 broader themes such as the impact of COVID-19 into spread and growth in cases, impact on economy and market, treatment and recovery, and impact on the health sector and governance response. Their result shows that average negative sentiments are seen on themes such as the growth of cases, whereas positive sentiments are seen on themes such as prevention, impact on the economy and market, government response, and treatment and recovery theme. Meanwhile, a public discourse and sentiment analysis of tweets related to COVID-19 in English language was analyzed using machine learning approaches by Xue et al. [29]. In their work, a total of eleven COVID-19-related topics were extracted using latent Dirichlet analysis (LDA) from all tweets collected between 23 January 2020 and 7 March 2020. Their result shows that the sentiment of fear is dominant in all topics.

Furthermore, Satu et al. [10] proposed a cluster-based classification and topic modeling (TClustVID), which first clusters the tweets into different clusters, each cluster containing positive, negative, and neutral classes. They performed classification using four classifiers such as decision tree, logistic regression, multilayer perception, and random forest. The evaluation results show that the second cluster produces the highest accuracy of 98.80% while comparing with baseline classifiers. Moreover, Aljameel et al. [14] conducted the sentiment analysis of COVID-19 based on tweets in the Arabic language. They investigated the uni-gram and bigram-based TF-IDF features with various classifiers such as SVM, KNN, and Naive Bayes. Their results show that the SVM classifier achieves the highest accuracy of 85% while using bigram TF-IDF-based features. Similarly, De et al. [30] performed the sentiment analysis of COVID-19 on tweets and the news article datasets in Brazil. A study on topic modeling and sentiment analysis of Brazilian text from news articles and tweets was presented in [30]. Their results show that both Twitter and news media provide similar kinds of information related to sentiment classification. Last but not the least, Ramya et al. [21] adapted logistic regression and Naive Bayes classifiers to analyze sentiments of COVID-19-related tweets into positive, negative, and neutral. Their result shows that logistic regression and Naive Bayes impart 91% and 74% accuracy, respectively. The sample summary of the performance of the few latest methods is presented in Table 1.

Considering that there are no well-established Nepali COVID-19 tweets' classification works conducted in the literature, we report some recent Nepali text/news document classification works in this study. Initially, Shahi et al. [31] classified Nepali documents using a support vector machine (SVM), which provides 74.65% accuracy. However, their method still has insufficient datasets for the evaluation. Similarly, Basnet and Timalsina [32] classified Nepali documents using the long short-term memory (LSTM) model, which provides 84.63% classification accuracy. Compared to Shahi et al., their method imparts a higher accuracy. However, their method still suffers from the problem of overfitting because of the lower amount of datasets. More recently, Sitaula et al. [1] proposed a supervised codebook approach and classified Nepali documents using a traditional machine learning classifier, called support vector machine (SVM), which reports 77.46%, 67.53%, 80.54%, and 89.58% accuracy on four different Nepali news datasets. Although they used four datasets in their study for the evaluation compared to other existing works, their method still suffers from the computational complexities triggered by the supervised codebook used in their work.

## 3. Materials and Methods

### 3.1. Dataset

We collect tweets from 11 Feb 2020 to 10 Jan 2021 using the geo-location of Nepal. To search the tweets on Twitter, we use only one keyword, called #COVID-19 (in the Nepali language). Each tweet is preprocessed and annotated by four annotators (co-authors) to set the sentiment labels using majority voting approach. The detailed statistics of our dataset is presented in Table 2.

### 3.2. Evaluation Metrics

We present the performance metrics used in our study. For the performance evaluation, we utilize widely popular metrics such as Precision (equation (1)), Recall (equation (2)), F1-score (equation (3)), and Accuracy (equation (4)):

(1) $$\begin{array}{c} P=\frac{\text{TP}}{\text{TP}+\text{FP}}, \end{array}$$

(2) $$\begin{array}{c} R=\frac{\text{TP}}{\text{TP}+\text{FN}}, \end{array}$$

(3) $$\begin{array}{c} F=2\times \frac{P\times R}{P+R}, \end{array}$$

(4) $$\begin{array}{c} A=\frac{\text{TP}+\text{TN}}{\text{TP}+\text{TN}+\text{FP}+\text{FN}}, \end{array}$$

where TP, TN, FP, and FN represent true positive, true negative, false positive, and false negative, respectively. Similarly, *P*, *R*, *F*, and *A* represent Precision, Recall, F1-score, and Accuracy, respectively.

### 3.3. Machine Learning Algorithms

We discuss eight traditional machine learning (ML) algorithms used in our work. They are support vector machine (SVM) with both linear and RBF (radial basis function) kernels, XGBoost (eXtreme gradient boosting), ANN (artificial neural networks), RF (random forest), NB (Naive Bayes), LR (logistic regression), and K-NN (K-nearest neighbors).

#### 3.3.1. Support Vector Machine (SVM)

Basically, the support vector machine (SVM) is a binary classifier [33], which learns to optimize a hyperplane defined in equation (5) using training data:

(5) $$\begin{array}{c} w.x-b=0, \end{array}$$

where *x* is a feature vector, *w* is a weight vector, and *b* is a bias. When the data are not linearly separable, the SVM uses kernel trick that implicitly maps the input features in another feature space (usually of higher dimension). The popular kernel functions used in various implementation of SVM are listed in equations (6)–(8) for linear, polynomial, and radial basis function (RBF) kernel, respectively [34]. Note that we use the linear and RBF kernel in this work, and classification results with these kernels are presented in Table 3.

(6) $$\begin{array}{c} K\left(x_{i},x_{j}\right)=\left\{x_{i}.x_{j}\right\}, \end{array}$$

(7) $$\begin{array}{c} K\left(x_{i},x_{j}\right)={\left(\gamma x_{i}.x_{j}+1\right)}^{d}, \end{array}$$

(8) $$\begin{array}{c} K\left(x_{i},x_{j}\right)=\exp\left(-\gamma {\left\|x_{i}-x_{j}\right\|}^{2}\right), \end{array}$$

where *K*(*x*_*i*_, *x*_*j*_) = *ϕ*(*x*_*i*_).*ϕ*(*x*_*j*_). Similarly, *d* and *γ* > 0 denote degree of polynomial and free parameter, respectively.

#### 3.3.2. XGBoost

XGBoost [35] is an ensemble-based tree boosting algorithm designed for large-scale machine learning applications. A group of weak learners are combined into strong learners using two methods: bagging and boosting. In gradient boosting technique, a new base learner is constructed in such a way that it will be maximally correlated with the negative gradient of the loss function with the whole ensemble in each iteration [36]. The XGBoost uses three kinds of boosting—gradient boosting, regularized boosting, and stochastic boosting—to surge the performance, reduce the computation time, and save the memory resources [37].

#### 3.3.3. Artificial Neural Network (ANN)

The artificial neural network is a combination of highly interconnected processing elements, known as neurons or nodes, aligned in three types of layers: one input layer, one or more hidden layers, and one output layer [31]. Each node represents a function that maps a weighted combination of input to activation of the neurons. An input vector is presented to the network, and its corresponding output is calculated. The weights are adjusted with optimization techniques such as “Adam,” “AdaGrad,” and “RMSProp” along with a backpropagation to compute the gradient of the loss function [38].

#### 3.3.4. Random Forest (RF)

Random forest is a popular learning algorithm that is based on the ensemble of decision trees with bagging approaches [39]. It starts with a decision tree by drawing a random sample of training data as a subset and creates a forest of decision tree classifiers. The size of the subsample is always the same, but the samples are drawn with replacement. A decision tree that is organized in the hierarchy is constructed through the binary partition starting from a root to a leaf node in the tree. Once the tree is fully formed, the validation data points traverse through the tree following a specific path and reach a leaf node that gives the corresponding output value. Finally, the output from the forest of trees is averaged to get the final output for a data point [40].

#### 3.3.5. Naive Bayes (NB)

A Naive Bayes classifier is based on the Bayes theorem of probability with strong independence assumptions between every pair of input features [41]. For input feature vector *x* = (*x*_1_,…, *x*_*n*_), given the class *y*, the estimation of probability distribution *P* (*x*_*i*_/*y*) in equation (9) defines the various types of Naive Bayes classifiers. For instance, multinomial Naive Bayes estimate the distribution parameters by a smoothed version of maximum likelihood or relative frequency counting. In this work, we use multinomial Naive Bayes implemented in Scikit-learn [34]:

(9) $$\begin{array}{c} P\left(y\;|\;x_{1},x_{2},\ldots ,x_{n}\right)=\frac{P\left(y\right)P\left(x_{1},x_{2},\ldots ,x_{n}\;|\;y\right)}{p\left(x_{1},x_{2},\ldots ,x_{n}\right)}. \end{array}$$

#### 3.3.6. Logistic Regression (LR)

It is an extension of the linear regression model for the classification problems [42]. Instead of fitting straight line as in linear regression, the logistic regression uses the function defined in equation (10) to squeeze the output between 0 and 1 as the probabilities:

(10) $$\begin{array}{c} \text{Logistic}\left(y\right)=\frac{1}{1+e^{-y}}. \end{array}$$

In this work, we use multinomial logistic regression with L2-regularization [43] as our COVID-19 tweets' sentiment classification is multiclass problem.

#### 3.3.7. K-Nearest Neighbor (K-NN)

K-nearest neighbor (KNN) is a nonparametric learning algorithm based on the simple but intuitive idea, where similar objects are within the closest proximity. It calculates the distance between a predefined number of training samples and the new query point to predict a label for a new point based on the majority. It is a kind of lazy learner that simply remembers all of its training data, and thus, it is nongeneralized. The common distance functions used are Euclidean distance, Manhattan distance, and Minkowski distance as defined in equation (11)–(13), respectively:

(11) $$\begin{array}{c} d_{e}=\sqrt{\overset{k}{\underset{i=1}{\sum }}{\left(x_{i}-y_{i}\right)}^{2}}, \end{array}$$

(12) $$\begin{array}{c} d_{m}=\overset{k}{\underset{i=1}{\sum }}\left|x_{i}-y_{i}\right|, \end{array}$$

(13) $$\begin{array}{c} d_{m}={\left(\overset{k}{\underset{i=1}{\sum }}{\left|x_{i}-y_{i}\right|}^{p}\right)}^{1/p}, \end{array}$$

where *p* represents the order of Minkowski distance and *x*_*i*_ and *y*_*i*_ represent two points on *k*-dimensional coordinate space.

### 3.4. Proposed Approach

In our method, we follow three different steps for the COVID-19-related tweets' sentiment classification, namely, “embedding vector extraction and representation,” “CNNs design and training,” and “decision fusion.”

### 3.5. Embedding Vector Extraction and Representation

Before extracting the embedding vector of each word in the tweets, we preprocess each raw token (or word) using the following method. First, we tokenize and remove alphanumeric characters from the each tweet. Second, we remove stop words using a rule-based approach. Last, we apply a Stemmer to attain the root word of each token. In summary, we follow a similar preprocessing approach as suggested in previous work [1].

For the extraction of the embedding vector of each clean token (*n*_*i*_), we adapt three different kinds of embedding vectors: fastText-based word embedding, domain-specific probability-based embedding, and domain-agnostic probability-based embedding. Here, feature selection is an important step in feature engineering to extract the discriminating features as suggested in [44]; however, we do not perform it in our work as our compact features already possess a lower-sized discriminating characteristic for the better classification.

First, we use fastText-based embedding vector (ft) [19], which has been pretrained with multilingual datasets [1]. This produces the contextual features based on the important clues related to each token. The size of the feature vector is 300-D. In this way, we represent each tweet as *n* × 300-sized matrix and perform average-pooling operation.

Second, we use the cross-domain dataset, Nepalinewsdataset [1], for the domain-agnostic probability-based (da) embedding vector extraction. This helps capture the cross-domain (non-COVID-19 related documents) information related to each token. For this, we first design the list of tokens, also called filterbank, for each category. Then, we calculate the probability of each token for each list as a feature value. For example, if there are 17 categories, the feature size of each token will be 17-D. In our work, Nepalinewsdataset has 17 categories, which, therefore, impart a 17-D sized feature vector for each token. This results in *n* × 17 matrix for each tweet, resulting in a 17-D vector after the average-pooling operation.

Third, we use the domain-specific probability-based approach (ds) to extract the embedding vector for each token as suggested by Sitaula et al. [1]. This helps capture the domain-specific (COVID-19 tweets' related) information corresponding to each token. Since our COVID-19 tweets' dataset has 3 classes, it provides a 3D feature vector for each token. In this way, we achieve each tweet as a matrix *n* × 3 tensor and then perform average-pooling operation.

### 3.6. CNNs' Design and Training

After the representation of each tweet, we design three different CNN models corresponding to each embedding type (“ft,” “ds,” and “da”). CNN models have been extensively used in different domains such as tweets' classification [45], scene image representation [46], remote-sensing image fusion [47], and biomedical image analysis [48]. It has produced a ground-breaking performance compared to the traditional approaches. With the help of several intermediate layers with convolution and pooling operations, it has been able to capture the discriminating information of several kinds of input data, including images and texts.

Here, we design simple, yet efficient, CNN models in our study. Three separate CNN models (equations (14)–(16)) are designed for fastText-based embedding (ft), domain-specific probability-based embedding (ds), and domain-agnostic-based embedding (da), respectively:

(14) $$\begin{array}{c} {\text{CNN}}_{\text{ft}}={\text{CNN}}_{\text{fastText}}\left(x\right), \end{array}$$

(15) $$\begin{array}{c} {\text{CNN}}_{\text{ds}}={\text{CNN}}_{\text{domainSpecific}}\left(x\right), \end{array}$$

(16) $$\begin{array}{c} {\text{CNN}}_{\text{da}}={\text{CNN}}_{\text{domainAgnostic}}\left(x\right), \end{array}$$

where *x*, CNN_ft_, CNN_ds_, and CNN_da_ denote the input tensor, CNN using fastText embedding, CNN using domain-specific probability embedding, and CNN using domain-agnostic probability embedding, respectively. The detailed architecture of each CNN used in our study is presented in Table 4.

### 3.7. Decision Fusion

We perform a fusion of decisions obtained from three different pretrained CNNs using ensemble CNN model for the end results (equation (17)). For the decision fusion using the ensemble CNN, we provide weights of 0.70, 0.20, and 0.10 empirically for CNN_ft_, CNN_da_, and CNN_ds_, respectively.

In our ensemble CNN model, we only unfreeze the top three layers of each fine-tuned CNN model and add the weighted decision fusion layer to attain the end results. The overall decision fusion pipeline of ensemble CNN is presented in Figure 2:

(17) $$\begin{array}{c} {\text{CNN}}_{c}=\text{Fusion}\left({\text{CNN}}_{\text{ft}},{\text{CNN}}_{\text{ds}},{\text{CNN}}_{\text{da}}\right), \end{array}$$

where CNN_*c*_ denote the fused CNNs' model using the weighted average method.

### 3.8. Implementation

For the implementation of our proposed method, we use two different tools, Sklearn [49] and Keras [50], implemented in Python [51]. Furthermore, we design 10 different train/test sets, each with 70 : 30 split ratio per category, and report the averaged performance measures over 10 runs for the analysis. To select the best hyperparameters in our study, we perform a grid search approach, which iterates over the range of different parameter values for the selection of optimal values. The detailed information of hyperparameters' selection approach for the corresponding ML algorithms is presented in Table 5.

## 4. Result and Discussion

### 4.1. Comparison of Proposed Feature Extraction Methods Using Traditional Machine Learning Methods

Here, we compare our proposed feature extraction methods based on traditional machine learning methods. The comparative results are presented in Table 3. While looking at Table 3, we notice that fastText-based embedding (ft) outperforms the other two embedding types (“ds” and “da”) in terms of Precision, Recall, F1-score, and Accuracy in most of the ML algorithms. For example, the XGBoost algorithm imparts 69.0%, 69.5%, 69.5%, and 66.7% for Precision, Recall, F1-score, and Accuracy, respectively. The performance superiority of “ft” among three methods is attributed to the compact contextual embedding vectors achieved from the pretrained fastText model, which has been trained with massive amount of Nepali documents. Similarly, the domain-specific (ds) embedding method is the second-best performing, which imparts a higher performance than the domain-agnostic (da) method on most of the ML algorithms. As an example, SVM + Linear imparts Precision of 63.5%, Recall of 54.1%, F1-score of 54.1%, and Accuracy of 56.3%. This interesting result reveals that the domain-specific (ds) information is very important to capture the domain-specific patterns of tweets. To this end, we are able to achieve prominent accuracy with a lower feature size (3-D). Finally, the domain-agnostic (da) method is the least performing, which has the lowest performance in most of the cases against two counterparts (“ft” and “ds”). We speculate that the reason of its lowest performance is responsible to the presence of less important contextual information.

While comparing different traditional machine learning methods on our proposed feature extraction techniques, we notice that the performance is differing from one ML algorithm to another algorithm. Under precision, SVM + RBF, RF, and SVM + Linear impart the highest performance on “ft” (70.2%), “da” (60.8%), and “ds” (63.5%), respectively. For Recall, XGBoost imparts the highest performance on “ft” (69.5%) and “ds” (62.3%), whereas RF yields the highest performance on “da” (60.7%). Under the F1-score, XGBoost imparts the highest performance on “ft” (69.5%) and “ds” (62.3%); however, RF imparts the highest performance on “da” (60.7%). Moreover, under accuracy, XGBoost imparts the highest performance on “ft” (66.7%) and RF imparts the highest performance on “da” (57.0%), whereas, on “ds” (65.7%) method, LR imparts the highest performance. Through this experiment, we stipulate that XGBoost is the high-performing algorithm in most cases as it can work on an optimal number of boosting trees, which could result in higher performance than its other counterparts.

Although the fastText-based method (ft) has the highest performance in comparison to other methods, it has a higher feature size (300-D) than other methods. Also, it is computationally infeasible to extract such features as we have to load pretrained models and compute them to achieve it. However, the second-best method (ds) has only a 3-D feature size and is easy to extract features. Achieving comparable performance with such a smaller-sized feature is an interesting research direction for future work.

### 4.2. Comparison of Our Methods with State-of-the-Art Methods

We compare our methods with the recent state-of-the-art methods [31, 32] and [1] that have been used for the classification of Nepali documents, particularly in news domain. We choose them because there are no existing works available in the literature for Nepali COVID-19 tweets' classification, and the available existing works in other languages such as English and Arabic are not appropriate to Nepali COVID-19 tweets' classification because of the different linguistic structure and processing requirements. To this end, we implement each method on our NepCOV19Tweets dataset and compare them with our proposed methods. The detailed experimental results are presented in Table 6.

While observing Table 6, we notice the superiority of our methods based on two different aspects. First, our proposed methods impart the comparable feature size, 3-D (ds), 17-D (da), 300-D (ft), and 320-D (ensemble CNN). Second, our methods impart the significant boost in the classification accuracy (68.7%), which has 9.2% improvement over the least-performing method (59.5%) and 5.8% improvement over the second-best method (62.9%). Such significant improvement of classification accuracy with a comparable feature size imparted by our methods has underlined the efficacy of domain-specific, domain-agnostic, and pretrained word embedding for the Nepali COVID-19 tweets' representation and classification.

### 4.3. Comparative Study of Proposed CNN Models Used in Our Study

We discuss the component analysis of each CNN model in terms of classwise performance. The results are presented in Table 7. Each CNN corresponds to three different kinds of features (“ft,” “ds,” and “da”) used in this study.

While looking at the performance of the fastText-based CNN model, called CNN_ft_, we notice that it provides an average accuracy of 68.1%, where it has the highest F1-score on the negative class and the lowest F1-score on neutral class. Similarly, the domain-specific CNN model (CNN_ds_) has the second-best performance (61.5% accuracy) among three components. It also imparts the highest F1-score on the negative class. We also notice a similar trend on CNN_da_, where it provides 59.5% accuracy with the highest performance on the Negative class (F1-score: 66.3%). Last but not the least, the ensemble of three CNN models (CNN_ft_, CNN_ds_, and CNN_da_) imparts an accuracy of 68.7%, which not only improves the overall performance but also outperforms each CNN models in this study.

In summary, the ensemble of three CNN models helps preserve three different semantic information in parallel for decision-making. This experiment further underscores that these three different pieces of information (“ft,” “ds,” and “da”) could play a crucial role in the discrimination of tweets during the sentiment classification process.

### 4.4. Statistical Analysis

Here, we perform the statistical analysis of performance measures (Precision, Recall, F1-score, and Accuracy). The results are presented in Figure 3. While looking at Figure 3, we notice that our method imparts 95% confidence interval (CI) of [67.8, 68.6], [68.3 68.9], [65.4 66.3], and [68.2 68.9] for Precision, Recall, F1-score, and Accuracy, respectively. We notice that the neutral class is complex compared to the positive and negative classes, which not only get a lower Precision and Recall measure but also contribute to a lower overall F1-score. Thus, we observe the slight degradation in the F1-score measure while looking at the box plot because of the neutral class. Moreover, while performing the two-tailed *t*-test, we notice that our method provides a *p* value < 2.2*e* − 16 for all performance measures (Precision, Recall, F1-score, and Accuracy). Because of such stable CI and significant two-tailed *t*-test results, we believe that our method is robust and prominent on sentiment classification for COVID-19-related tweets.

## 5. Conclusion and Future Works

In this paper, we have proposed three CNN models to classify the Nepali COVID-19-related tweets into three sentiment classes (positive, negative, and neutral). These CNN models show stable and robust performance. Also, we have proposed to use three different kinds of feature extraction methods for the representation of tweets during classification. We have validated our proposed features' extraction methods using traditional machine learning algorithms, which show that our proposed features can discriminate the complex COVID-19 tweets in most cases.

Our method has three main limitations. First, our method ignores the sequential approach of tokens, which could be an important clue for tweets classification. To this end, the sequential-based model such as the LSTM (long short-term memory) model could contribute to the performance improvement. Second, our method exploits fastText (“ft”) and probability-based embeddings (“ds” and “da”) for the classification. The combination of other kinds of embeddings such as Word2vec and GloVe could enhance the performance further.

## Figures and Tables

**Figure 1:** Nepali alphabets and numerals [1].

**Figure 2:** Decision fusion using weighted average method on ensemble CNN (CNN_*e*_).

**Figure 3:** Statistical analysis of performance measures over results of 10 folds used in our study.

**Table 1:** Summary performance (%) of sentiment classification of some state-of-the-art methods on tweets.

Method	Dataset	Accuracy (%)	Methodology	Limitations
Basir et al. [8]	StanfordSentiment140 [8]	85.4	(i) Stacked ensemble method	(i) Ignore the effects of global COVID-19 news on sentiment analysis beside the specific country
Rustam et al. [7]	Covid-19Tweets [20]	93.0	(ii) BoW with various ML methods	(ii) Limited performance on small datasets
Aljameel et al. [14]	Self-created dataset	85.0	(iii) N-gram with various ML methods	(iii) Feature selection and hyperparameter tuning operation is not performed
Ramya et al. [21]	Self-created dataset	91.0	(iv) Naive Bayes	(iv) Experimented with a limited data
Naseem et al. [5]	COVIDSenti [5]	92.2	(v) ML methods such as Naive Bayes, support vector machine, and random forest	(v) Limited to English tweets
Satu et al. [10]	Covid-19Tweets [20]	98.8	(vi) Cluster-based classification	(vi) Tweets search limited to a few keywords in English text

**Table 2:** Our NepCOV19Tweets dataset statistics.

Class	No. of raw tokens	No. of raw tweets	No. of clean tokens	No. of clean tweets
Positive	291,593	14,982	198,504	14,957
Neutral	85,175	4860	55,679	4744
Negative	247,548	13,593	162,669	13,546
Total	624,316	33,435	416,852	33,247

**Table 3:** Comparison of our method with existing machine learning algorithms in terms of classification performance (%).

Algorithms	Ft				da				ds			
	*P*	*R*	*F*	*A*	*P*	*R*	*F*	*A*	*P*	*R*	*F*	*A*
SVM + Linear	67.1	62.2	62.2	63.9	57.3	44.0	44.0	47.2	**63.5**	54.1	54.1	56.3
SVM + RBF	**70.2**	51.0	51.0	40.2	58.5	53.9	53.9	55.5	63.2	51.5	51.5	54.6
XGBoost	69.0	**69.5**	**69.5**	**66.7**	58.3	59.8	59.8	56.3	61.5	**62.3**	**62.3**	58.9
ANN	63.1	63.7	63.7	63.4	56.8	58.8	58.8	54.7	62.0	61.9	61.9	58.0
RF	69.6	67.5	67.5	63.5	**60.8**	**60.7**	**60.7**	**57.0**	59.9	61.9	61.9	59.5
NB	59.4	56.1	56.1	57.5	47.0	48.7	48.7	44.9	48.5	50.0	50.0	45.8
LR	65.1	67.4	67.4	64.7	54.2	56.6	56.6	52.0	63.2	61.8	61.8	**61.8**
K-NN	65.2	65.2	65.2	60.3	51.8	57.5	57.5	52.8	61.3	61.6	61.6	57.4

Note that *P*, *R*, *F*, and *A* denote overall Precision, Recall, F1-score, and Accuracy for three types of embeddings (ft: fastText, da: domain-agnostic, and ds: domain-specific), respectively. The hyperparameters of traditional machine learning algorithms are as follows: SVM + Linear (*c*: 1, Gamma: 0.1), SVM + RBF (*c*: 100, Gamma: 0.1), XGBoost (learning-rate: 0.1, max-depth: 7, *n*-estimators: 150), ANN (Hidden-layer-size: 20, learning-rate-init: 0.01, max-iter: 1000), RF (min-sample-leaf: 3, min-sample-split: 6, *n*-estimators: 200), LR (*C*: 10, solver: lbfgs, max-iter: 1000), and K-NN (leaf-size: 35, *n*-neighbor: 120, p: 1). Boldface denotes the highest performance.

**Table 4:** The architecture of three CNNs proposed in our work.

Layer	CNN_da_		CNN_ds_		CNN_ft_	
	(*n*, *s*)	Output shape	(*n*, *s*)	Output shape	(*n*, *s*)	Output shape
Input	—	(17, 1)	—	(3, 1)	—	(300, 1)
Conv1D + Relu	(32, 3)	(15, 32)	(8, 2)	(2, 8)	(32, 3)	(298, 32)
Conv1D + Relu	(16, 3)	(13, 16)	(8, 2)	(1, 8)	(16, 3)	(296, 16)
Flatten + Dropout (0.2)	—	208	—	8	—	4736
Dense + Dropout (0.2)	—	128	—	6	—	128
Dense	—	64	—	4	—	64
Softmax	—	3	—	3	—	3

Note that (*n*, *s*) denotes the number of filters and filter size for the corresponding CNN model.

**Table 5:** Grid search ranges used to tune the corresponding hyperparameters of each machine learning algorithm used in our study.

Algorithm	Range
SVM + Linear	*C*: {1 to 1000}, Gamma: {0.001 to 0.1}
SVM + RBF	*C*: {1 to 1000}, Gamma: {0.001 to 0.1}
XGBoost	Learning-rate: {0.01 to 0.1}, max-depth: {5 to 10}, *n*-estimators: {120 to 200}
ANN	Hidden-layer-size: {20 to 60}, learning-rate-init: {0.01 to 1}, max-iter: {10 to 1000}
RF	Min-sample-leaf: {3 to 7}, min-sample-split: {2 to 6}, *n*-estimators: {50 to 200}
LR	*C*: {1 to 1000}, solver: lbfgs, max-iter: {100 to 1000}
K-NN	Leaf-size: {30 to 45}, *n*-neighbor: {100 to 200}, *p*: {1 to 3}
Our CNN models	Learning-rate: {1*e* − 01, 1*e* − 02, 1*e* − 03, 1*e* − 04, 1*e* − 05}, batch-size: {8, 16, 32, 64}, epochs: {10, 20, 30, 40, 50, 100}, optimizer: {“RMSProp”, “Adam,” “SGD”}

**Table 6:** Comparison of our methods based on overall classification accuracy (%) with state-of-the-art methods.

Methods	Feature size	Accuracy
Shahi et al. [31]	100-D	62.1
Basnet and Timalsina [32]	300-D	62.9
Sitaula et al. [1]	17-D	59.8
Ours (ds)	3-D	61.5
Ours (da)	17-D	59.5
Ours (ft)	300-D	68.1
Ours (ensemble)	320-D	68.7

Note. Each reported accuracy in the table is the averaged value over 10 runs on our NepCOV19Tweets dataset.

**Table 7:** Classwise study of our proposed method using classification performance (%).

CNN	Positive			Neutral			Negative			Overall			
	*P*	*R*	*F*	*P*	*R*	*F*	*P*	*R*	*F*	*P*	*R*	*F*	*A*
CNN_ft_	69.4	**74.6**	71.8	51.8	**22.4**	**31.1**	**69.5**	76.8	72.8	63.5	**57.9**	**58.5**	68.1
CNN_ds_	68.0	59.6	62.6	12.7	00.2	00.5	59.0	82.7	68.6	46.5	47.5	43.9	61.5
CNN_da_	64.1	57.6	60.5	43.9	04.5	08.2	57.4	78.6	66.3	55.1	46.9	45.0	59.5
CNN_*c*_	**71.8**	72.0	**71.9**	**63.0**	14.7	23.7	66.8	**82.7**	**73.8**	**67.2**	56.4	56.4	**68.7**

Note/ *P*, *R*, and *F* denote Precision, Recall, and F1-score for three classes (positive, negative, and neutral), respectively. Note that the hyperparameters used in our models are as follows: learning-rate: 1*e* − 05, batch-size: 32, epochs: 50, and optimizer: RMSProp. Boldface denotes the highest performance.

## Data Availability

Data and source code used to support the findings of the study are available from the corresponding author upon request.
